The article "Using a Random Forest Model to Study the Impact of Local Government-Led Urbanization on Urban Sustainable Development" was published in 2022. Journal: J Environ Public Health.

# Using a Random Forest Model to Study the Impact of Local Government-Led Urbanization on Urban Sustainable Development

**DOI:** 10.1155/2022/3393532

**Published:** 2022-07-06

**Authors:** Yixiao Peng

**Affiliations:** School of Economics, Zhejiang University of Technology, Hangzhou 310023, Zhejiang, China

## Abstract

Urbanization has accelerated China's economic growth, but it has also brought many sustainability issues. This paper selected a random forest model to study the impact of local government-led urbanization on urban sustainable development. Urbanization affected urban sustainable development through government revenue expansion, land resources mismatch, and industrial structure adjustment. The results showed that the adjustment of industrial structure has the greatest impact on urban sustainable development, and the importance of the average output of industrial enterprises confirms it. Government revenue expansion and land resources mismatch are more important to the sustainable development of representative urban agglomerations. The goodness of fit of the random forest model is better than the multiple linear regression (MLR) model and the extreme gradient boosting (XGBoost) model. The generalization ability of the model is improved with the optimization of variables. The main contribution of this paper is that we have established a complete information dynamic game model on government revenue expansion, land resource mismatch, industrial structure adjustment, and urban sustainable development. And the random forest model is used to study the relationship between the above variables.

## 1. Introduction

In the current stage of China's urbanization process, land resource mismatch, imbalance of industrial structure, and government revenue expansion have brought negative impacts on the urban sustainable development. China's central government has regarded GDP development as the primary goal in the past, and it regards achievements in GDP development as the promotion standard of local government officials [1]. Promotion incentives enable local governments to accelerate economic development through land management [2].

There are three mechanisms for local governments to develop the economy through land management. Firstly, local governments attract enterprises and residents to invest in urban construction through the land resources mismatch. As the local governments control the supply of the primary land market, the price of commercial residential land is much higher than that of industrial land [3–5]. The low price of industrial land has attracted enterprise investment, while the increasing price of commercial and residential land has attracted residents to invest in real estate; these investments boost economic growth [6, 7]. However, local governments attract investment through low-price competition, and the cheap industrial land lowers the entry threshold for companies, resulting in excess capacity and environmental pollution [8–10].

The article "Using a Random Forest Model to Study the Impact of Local Government-Led Urbanization on Urban Sustainable Development" was published in 2022. Journal: J Environ Public Health.

Secondly, local governments have gained more revenue through the price difference between industrial land and commercial residential land to promote economic growth, which is called land finance [11–13]. In the long-term process of developing the economy by operating land, the local government has become dependent on land finance and increased its income by continuously hoarding land and raising the price of land [7, 14]. This approach has created a speculative bubble in the real estate market, which is not sustainable. At the same time, land finance has also caused many unsustainable problems such as environmental pollution and increased carbon emissions [15–17].

Thirdly, land development led by local governments accelerates urbanization and increases the rate of economic growth [18–20]. Land development expands urban areas and promotes economic growth through capital accumulation [21–23]. Urbanization concentrates population density and increases the ecological footprint, pushing the environment beyond carrying capacity [24–26]. In the process of industrialization, urbanization, and economic development, urban carbon emissions have increased significantly [27–31]. Some local governments blindly promote urbanization to develop the economy, resulting in many ghost towns [32]. The excessive urban expansion will also occupy many arable land resources, thus threatening the ecological environment and sustainable development [23, 33–35].

In general, urbanization, economic development, and land management led by the government will bring environmental problems, which have seriously hindered urban sustainable development. However, sustainable development involves more than just the environmental dimension; the Sustainable Development Goals system (SDGs) projected by the United Nations covers seventeen areas such as good health, quality education, and economic growth. As urbanization, land resources mismatch, and economic development bring more government revenue, China's sustainable development elements such as infrastructure, living standards, and public services have greatly improved [36–40]. Therefore, the urbanization led by the government will affect the level of urban sustainable development, and the direction of urban sustainable development depends on government expenditure preferences and land development planning. If local governments intend to channel revenues more to growth-oriented infrastructure, it will crowd out expenditure on welfare programs and public services [41]. Infrastructure investment will further increase government revenue and form internal strengthening mechanisms [42, 43], which cause excessive urbanization and hinder urban sustainable development. If the local government provides more land for the construction of public services and intends to channel revenues more to industrial restructuring, the living conditions of residents will be improved, and environmental pollution and carbon emissions will be reduced [44, 45].

The article "Using a Random Forest Model to Study the Impact of Local Government-Led Urbanization on Urban Sustainable Development" was published in 2022. Journal: J Environ Public Health.

The contributions of this paper can be summarized as follows: (1) The complete information dynamic game model we build shows a new theory about government revenue expansion, land resources mismatch, industrial structure adjustment, and urban sustainable development. (2) The random forest model was selected to fit the nonlinear relationship between government revenue expansion, land resources mismatch, industrial structure adjustment, and urban sustainable development. (3) More detailed conclusions are drawn from the study of the eastern, central, and western representative urban agglomerations.

In the rest of this paper, the second section introduces the theoretical model; the third section introduces methodology and data; the fourth section shows the results and discussion; the fifth section gives the conclusions.

## 2. Theoretical Model

The promotion incentive mechanism makes local governments compete in revenue expansion, urbanization, land management, and industrial development. This competition can be described as a simple Nash equilibrium game (Table 1). Suppose that local government A and local government B have two strategies of GDP development and sustainable development. Both strategies can make local governments obtain the payoff of regional GDP level improvement *ρ* and government revenue increases *σ*. The local government will develop strategies based on the total payoff *ρ*+*σ*. Under the economic development strategy, local governments channel revenues more to growth-oriented infrastructure, which promotes GDP growth, accelerates the process of urbanization, and brings additional revenue. As the sustainable development strategy requires the government to invest revenue in public services and industrial upgrading, this will slow down urbanization and economic growth and cause *ρ*, *σ*_1_ > *σ*_2_. Therefore, local governments that adopt the GDP development strategy can always obtain more payoffs. In the equilibrium state, local governments A and B will adopt the GDP development strategy, which maximizes the payoff for both sides.

However, the development of GDP with the realization of sustainable economic development is not achieved overnight, and industrial upgrading is a long process. The above Nash equilibrium cannot accurately reflect the game relationship of local governments. Therefore, this study introduces the complete information dynamic game model to demonstrate the game relationship between local governments [46].

The article "Using a Random Forest Model to Study the Impact of Local Government-Led Urbanization on Urban Sustainable Development" was published in 2022. Journal: J Environ Public Health.

On the premise of completely taking economic development as the goal, the utility function of local government can be expressed as

(1) $$\begin{array}{c} U_{i}=\beta x_{i}+\theta_{1}y_{i}-z_{i}. \end{array}$$

*U*_*i*_ is the total utility of local government. *x*_*i*_ represents the revenue scale of local governments (including general public budget revenue, social insurance revenue, and land revenue). Urbanization will promote economic development and increase government revenue. *β* is the marginal utility of government revenue, including public services, infrastructure investment to stimulate economic growth, making up the deficit, and official promotion. *y*_*i*_ is GDP. *θ*_1_ is the marginal utility of GDP development. *z*_*i*_ is the negative impact of economic development and urbanization, such as arable land degradation, environmental pollution, and overcapacity.

Since the central government has put forward the goal of sustainable development, we assume that local governments choose industrial upgrading with a ratio *α*. *θ*_2_ is the marginal utility of industrial upgrading. The size of *θ*_1_ and *θ*_2_ depends on the development strategy of the central government. The utility function of local government can be expressed as

(2) $$\begin{array}{c} U_{i}=\beta \left(1-\alpha \right)x_{i}+\theta_{1}\left(1-\alpha \right)y_{i}-z_{i}+\theta_{2}\alpha y_{i}. \end{array}$$

Industrial upgrading needs government support, so the government revenue is reduced to (1 − *α*)*x*_*i*_. The competition between local governments will produce negative spillover effects, and the actual utility of local governments 1 and 2 can be expressed as

(3) $$\begin{array}{c} U_{1}^{\prime }=U_{1}-\gamma_{1}U_{2}, \end{array}$$

(4) $$\begin{array}{c} U_{2}^{\prime }=U_{2}-\gamma_{2}U_{1}. \end{array}$$

The relationship between *U*_1_′ and *α*_1_ can be expressed as

(5) $$\begin{array}{c} \frac{\text{d}U_{1}^{\prime }}{\text{d}\alpha_{1}}=-\beta x_{1}-\left(\theta_{1}-\theta_{2}\right)y_{1}. \end{array}$$

When *θ*_1_ > *θ*_2_ and d*U*_1_′/d*α*_1_ < 0, reducing the industrial upgrading ratio *α*_1_ will increase the actual utility of local government 1. The relationship between *U*_1_′ and *α*_2_ can be expressed as

(6) $$\begin{array}{c} \frac{\text{d}U_{1}^{\prime }}{\text{d}\alpha_{2}}=\gamma_{1}\left[\beta x_{2}+\left(\theta_{1}-\theta_{2}\right)y_{2}\right]. \end{array}$$

When *θ*_1_ > *θ*_2_*θ*_1_ > *θ*_2_ and (d*U*_1_′/d*α*_2_) > 0, reducing industrial upgrading ratio *α*_2_ will reduce the actual utility of local government 1. Equations (5) and (6) show that if the local government pays more attention to GDP development, reducing the industrial upgrading ratio will increase its own actual utility and reduce the actual utility of other local governments. This will lead local governments to abandon the industrial upgrading strategy and join the GDP development competition.

The article "Using a Random Forest Model to Study the Impact of Local Government-Led Urbanization on Urban Sustainable Development" was published in 2022. Journal: J Environ Public Health.

However, as the local government revenue rises rapidly, the central government will penalize this behavior to protect the economy, and it leads to *β* < 0. If the penalization is sufficiently severe, equations (5) and (6) will be less than 0. Local government 1 will increase the industrial upgrading ratio *α*_1_ to improve its own actual utility, and it will reduce the actual utility of local government 2.

Government expenditure cannot permanently stimulate the GDP development, and urbanization also has bottlenecks, so we assume that *x*_*i*_ and *y*_*i*_ have the following function:

(7) $$\begin{array}{c} y_{i}=c\;\ln\;x_{i}. \end{array}$$

Studies have proved that China's carbon emissions, environment, and other sustainable development factors have Kuznets Curve [47–49]. We assume that *z*_*i*_ and *y*_*i*_ have the following function:

(8) $$\begin{array}{c} z_{i}=ay_{i}-by_{i}^{2}. \end{array}$$

*a*, *b*, and *c* are positive parameters. Taking equations (7) and (8) into equation (6),

(9) $$\begin{array}{c} U_{i}=\beta \left(1-\alpha \right)x_{i}+\theta_{1}\left(1-\alpha \right)c\;\ln\;x_{i}-\left(a\left(1-\alpha \right)c\;\ln\;x_{i}-b{\left(1-\alpha \right)}^{2}c^{2}{\left(\ln\;x_{i}\right)}^{2}\right)+\theta_{2}\alpha c\;\ln\;x_{i}. \end{array}$$

The first-order condition can be obtained by taking the derivative of *x*_*i*_:

(10) $$\begin{array}{c} \frac{\text{d}U_{i}}{\text{d}x_{i}}=\beta \left(1-\alpha \right)+\left[\left(\theta_{1}-\theta_{2}-a\right)\left(1-\alpha \right)+\theta_{2}+\;2b{\left(1-\alpha \right)}^{2}c\;\ln\;x_{i}\right]\frac{c}{x_{i}}. \end{array}$$

When *β* > 0, if *θ*_1_ − *θ*_2_ > *a*, (d*U*_*i*_/d*U*_*i*_) > 0. It shows that when the marginal utility of GDP development is bigger than that of industrial upgrading, the local government will improve its own utility by expanding the scale of government revenue. However, as *x*_*i*_ increases large enough, the second term on the right of equation (10) approaches 0, and the symbol d*U*_*i*_/d*U*_*i*_ depends on the financial supervision strategy of the central government *β*. If the central government takes punitive measures (*β* < 0), local governments will decrease their revenue. If the central government chooses to ignore (*β* > 0), local governments will continue to increase the scale of revenue.

The article "Using a Random Forest Model to Study the Impact of Local Government-Led Urbanization on Urban Sustainable Development" was published in 2022. Journal: J Environ Public Health.

Equation (10) can be transformed as

(11) $$\begin{array}{c} \frac{\text{d}U_{i}}{\text{d}x_{i}}=\left(1-\alpha \right)\left[\beta +2b\left(1-\alpha \right)\frac{c^{2}}{x_{i}}\ln\;x_{i}\right]+\left[\theta_{1}\left(1-\alpha \right)+\alpha \theta_{2}-a\left(1-\alpha \right)\right]\frac{c}{x_{i}}. \end{array}$$

If ∀*x*_*i*_, there is d*U*_*i*_/d*x*_*i*_ < 0, then *β*, *θ*_1_, and *θ*_2_ need to satisfy two conditions. Firstly, *β* < −[2*b*(1 − *α*)*c*^2^ln  *x*_*i*_]/*x*_*i*_*β* < −[2*b*(1 − *α*)*c*^2^ln  *x*_*i*_]/*x*_*i*_; it means that the marginal utility of government revenue is negative, and the central government has strengthened financial supervision. Secondly, *θ*_1_ < −[*α*/(1 − *α*)*θ*_2_]*θ*_1_ < −[*α*/(1 − *α*)*θ*_2_]; it means that the marginal utility of GDP government is negative, and local government will choose the industrial upgrading strategy. These two conditions are indispensable. If the GDP development encounters a bottleneck and the central government chooses a loose financial supervision strategy, local governments will still maintain GDP growth by expanding the scale of government revenue. This will lead to unsustainable problems such as land resources mismatch and overcapacity; if the GDP development lags behind and the central government chooses a strict financial supervision strategy, the development enthusiasm of local governments will be reduced. Insufficient fiscal revenue will prevent local governments from providing adequate public services such as healthcare and education.

For the central government, the increase in revenue can improve the level of public facilities such as national defense, infrastructure, medical care, and education and promote economic growth to improve people's living standards. For local governments, the increase in fiscal revenue can achieve the GDP target set by the central government and reduce the deficit. However, development aimed at increasing fiscal revenue has drawbacks. In pursuit of the dual goals of GDP scale and government revenue scale, high pollution and high energy consumption have appeared, and this phenomenon has entered a vicious circle.

In general, the financial supervision strategy and economic development strategy of the central government will affect the decision-making of local governments in industrial structure adjustment and revenue adjustment. Different development stages should correspond to different strategies. In the early stage of economic development, the central government adopts a loose fiscal supervision strategy and a GDP development strategy, and local governments can increase government revenue through the land resources mismatch to develop GDP and provide more public services. As the GDP development encounters bottlenecks, the central government should adopt a strict financial supervision strategy and a sustainable development strategy, and local governments should reduce government revenue, adjust industrial structure, and solve the problem of land resources mismatch.

The article "Using a Random Forest Model to Study the Impact of Local Government-Led Urbanization on Urban Sustainable Development" was published in 2022. Journal: J Environ Public Health.

As China's GDP growth rate declines, the government needs to actively change the way of economic development. Local governments should not rely on developing GDP by land management, especially for the land resources mismatch. Researches show that land transfer marketization can improve the industrial structure and reduce environmental pollution [50–52]. Therefore, local governments should make efforts to control the scale of government revenue, reduce the investment in growth-oriented infrastructure, provide more public services, and support industrial upgrading.

## 3. Methodology and Data

### 3.1. Urban Sustainable Development Index (USDI)

#### 3.1.1. Indicators Selection

Studies on sustainability measurement are mainly based on provincial data [53–55]. Based on the perspective of land resources mismatch, the competition between local governments is more obvious. Therefore, this study attempts to measure the level of urban sustainable development. However, multidimensional evaluation can accurately calculate the level of urban sustainable development. However, due to the limited integrity of urban data, we comprehensively consider the integrity and diversity of the data. The basis of data selection is as follows: Firstly, refer to the SDGs sustainable index evaluation system. Secondly, select widely used indicators. Thirdly, select representative indicators. Finally, we have selected 7 indicators to form an urban sustainable development index (Table 2).

The indicators cover three aspects of economy, society, and environment. All indicators include 292 city data from 2000 to 2019. The carbon emissions data were obtained from the research of Chen [56]. Other data were obtained from the China Urban Statistical Yearbook. The missing data are supplemented by the interpolation method.

#### 3.1.2. Calculation

All indicators need to be normalized to eliminate dimensional discrepancies, and the normalization equations are as follows:

(12) $$\begin{array}{c} x^{\text{'}}=\frac{x-x_{\text{min}}}{x_{\text{max}}-x_{\text{min}}}, \end{array}$$

(13) $$\begin{array}{c} x^{\text{'}}=\frac{x_{\text{max}}-x}{x_{\text{max}}-x_{\text{min}}}. \end{array}$$

Equations (12) and (13) apply to positive and negative indicators, respectively; the standardized indicators are within the interval [0, 1]. However, the geometric mean method with a standardized indicator of zero would result in an SDI of zero. We need to set a minimum value to ensure that all standardized indicators are within the interval (0, 1]. The upper limit also needs to be set for indicators of sustainable development.

The article "Using a Random Forest Model to Study the Impact of Local Government-Led Urbanization on Urban Sustainable Development" was published in 2022. Journal: J Environ Public Health.

The USDI is established using the geometric mean method with reference to the method of the Human Sustainable Development Index (HSDI) [57, 58]. The calculation formula is as follows:

(14) $$\begin{array}{c} \text{USDI}=\sqrt[{7}]{\prod_{i=1}^{7}x_{i}}. \end{array}$$

*x*_*i*_ is the value of the indicator after normalization. The reason for using the geometric mean calculation is that there should be a nonlinear substitution relationship between indicators, and the geometric mean method can penalize cities with unbalanced development [59–61].

### 3.2. Selection of Explanatory Variables

Explanatory variables include industrial structure (IS), government revenue level GR(GR), and degree of land resources mismatch (LRM). The proportion of the tertiary industry GDP in different cities in China varies greatly, so the proportion of GDP of the tertiary industry is used to represent the industrial structure.

The government revenue level is represented by the ratio of local government revenue to GDP. Local government revenue includes local governments' general public budget revenue (GPBR), social insurance funds revenue (SIFR), and land revenue (LR).

Land transfer methods in China include agreement, tenders, auction, and listing transfers. Tenders, auctions, and listings for sale can get higher unit prices due to the market-oriented transfer. Therefore, the government will use the lower-priced agreement land to attract investment and then transfer the higher-priced tender auction and listing land to commercial and residential real estate. This way of selling is called land resources mismatch. Firstly, it can develop GDP by attracting investment; secondly, it can increase the local government revenue by raising the market price of land. In summary, the degree of land resources mismatch can be expressed as follows:

(15) $$\begin{array}{c} {\text{LRM}}_{\text{it}}=\left\{\begin{array}{cc} \frac{{\text{AGR}}_{\text{it}}}{{\text{TAL}}_{\text{it}}}, & {\text{LRM}}_{\text{it}}\leq 1,\\ 1, & {\text{LRM}}_{\text{it}}>1. \end{array}\right. \end{array}$$

AGR_it_ is the unit prices of agreement transfer, and TAL_it_ is the unit prices of tender, auction, and listing transfer. As there is a correlation between annual land revenue and the unit price gap, we believe that the unit price ratio is more suitable for measuring the degree of land resource mismatch than the area ratio, which is different from existing research methods [10, 62]. Normally, land buyers refuse to bear the premium, but due to the small scale of land transfer in some cities, there are special agreements for sales in some years that cause AGR_it_>TAL_it_. Therefore, when LRM_it_ > 1, it means that there is no land resources mismatch.

The article "Using a Random Forest Model to Study the Impact of Local Government-Led Urbanization on Urban Sustainable Development" was published in 2022. Journal: J Environ Public Health.

Since there are many factors affecting the level of sustainable development, the absence of variables will cause regression bias. Therefore, auxiliary variables need to be added to improve the goodness of fit of the model, which can improve the prediction accuracy of the model. We attempted to add population density (PD), geographic location (GL), real estate development level (RED), and average output of industrial enterprises (AOIE) as auxiliary explanatory variables. All these factors will affect the government's decision-making in urban sustainable construction. For example, the local government will plan the number of hospitals and schools based on the city's population density; the local government will plan the proportion of residential, commercial, and industrial land for the next year based on the real estate development situation; the local government will decide whether to close polluting enterprises based on the urban environment. However, adding auxiliary explanatory variables does not necessarily improve the accuracy of the model because the added variables may not be relevant to urban sustainability. We can select the variables based on which combination performs better. If the added variables did not improve the goodness of fit of the model, we chose to ignore these variables.

IS, GPBR, PD, RED, and AOIE data are from China Urban Statistical Yearbook. SIFR data are from China Statistical Yearbook. LR, AGR, and TAL data are from China Land Resources Statistical Yearbook.

### 3.3. Machine Learning Method-Random Forest

The random forest model is a kind of machine learning method proposed by Breiman [63]. It consists of multiple decision trees, and each decision tree is independent (Figure 1).

The random forest model is an ensemble learning and bootstrap sampling process; suppose the original sample set contains *N* samples and *M* features. Firstly, for each decision tree, repeatedly and randomly select *N* samples from the original sample set with replacements to generate a new training sample set. Repeated sampling will cause some samples not to participate in the splitting of the decision tree, which is called out of bag (OOB). OOB is used to estimate the misclassification rate of decision trees. For each node of the decision tree, randomly select *m* features as the split basis (*m* ≪ *M*). Secondly, using the Classification and Regression Tree (CART) with algorithm regressing each tree, the objective function is as follows:

(16) $$\begin{array}{c} \min\sum_{j=1}^{J}\sum_{i\in R_{j}}{\left(y_{i}-{\hat{y}}_{R_{j}}\right)}^{2}. \end{array}$$

*R*_*j*_ represents dividing the sample into *j* distinct regions, and ${\hat{y}}_{R_{j}}$ represents the average predicted value in *R*_*j*_. Different from the traditional CART algorithm, the random forest model requires the decision trees split completely and ensure the integrity of the trees. Thirdly, take the average of all decision tree predictions as the prediction result of the random forest model. Model prediction accuracy is evaluated by root mean squared error (RMSE) and goodness of fit (*R*^2^).

The article "Using a Random Forest Model to Study the Impact of Local Government-Led Urbanization on Urban Sustainable Development" was published in 2022. Journal: J Environ Public Health.

The reasons for choosing the random forest model in this study were as follows: (1) Studies have shown that the relationship between urban development, land resource allocation, and sustainability factors such as air quality, carbon emissions, and environmental pollution is nonlinear. Due to the antioverfitting and antinoise capabilities, the random forest model is widely used in the study of nonlinear problems [64–70]. (2) The construction decision-making process of local governments in urbanization is similar to decision trees in random forests. For example, when land resources are expropriated, how many hospitals should be planned? Hundreds of local governments will make decisions based on urban conditions (Figure 2), and the mean value of local government plans in similar cities is the predicted value.

To improve the accuracy of the prediction results, we use three models for random forest regression. Model 1 is the base model, consisting of USDI, GR, LRM, and IS:

(17) $$\begin{array}{c} \text{USDI}∼\text{GR}+\text{LRM}+\text{IS.} \end{array}$$

Model 2 adds PD, GL, RED, and AOIE, supplementing other factors affecting sustainable development in the process of urbanization:

(18) $$\begin{array}{c} \text{USDI}∼\text{GR}+\text{LRM}+\text{IS}+\text{PD}+\text{GL}+\text{RED}+\text{AOIE.} \end{array}$$

Model 3 splits the GR to study the impact of different revenues on USDI:

(19) $$\begin{array}{c} \text{USDI}∼\text{GPBR}+\text{SIFR}+\text{LR}+\text{LRM}+\text{IS}+\text{PD}+\text{GL}+\text{RED}+\text{AOIE.} \end{array}$$

Extreme gradient boosting model (XGBoost) and multiple linear regression (MLR) will be used to test the robustness of all models.

## 4. Results and Discussion

### 4.1. Predictive Performance of Random Forest Model

We divide the original sample into two parts: 70% of the data are used for training, and 30% of the data are used for testing. The training set is used for model regression, and the testing set is used to examine the generalization ability of the model.

The article "Using a Random Forest Model to Study the Impact of Local Government-Led Urbanization on Urban Sustainable Development" was published in 2022. Journal: J Environ Public Health.

Table 3 shows that *R*^2^ of the base model on the test set is only 45.9%. By adding auxiliary explanatory variables, *R*^2^ of the test set can be improved to 70.4%. Further splitting the GR improves *R*^2^ of the test set to 74.0%. Compared with the split of GR, the auxiliary explanatory variables have a greater improvement in the fit of the prediction set. The addition of auxiliary explanatory variables significantly improves the generalization ability of the model and reduces the dispersion of the prediction set (Figure 3). The robustness test (Table 3) shows that the performance of the random forest model is better than that of XGboost or MLR.

Figure 4 shows the importance of variables in a different model. In the base model, GR has the highest importance. After adding auxiliary explanatory variables, IS becomes the most important variable in model, indicating that the synergy of AOIE and IS has a higher impact on sustainable development than GR. The increase of AOIE and IS will reduce the discharge of industrial wastewater and exhaust gas, which will affect the USDI. After the split of GR, the importance of LRM has increased, probably because of the synergistic effect with LR. Local governments will increase the LR by changing the LRM strategy. The importance of AOIE decreases, while the importance of SIFR is similar to that of AOIE. SIFR is highly correlated with the number of hospitals and schools, and AOIE is highly correlated with industrial wastewater and air emissions, so both have the same impact on USDI. PD and GL both have great importance to USDI, which has not changed before or after splitting GR. Urbanization will increase the number and density of urban populations, and local governments will improve healthcare and education. China's eastern cities have more permanent residents than registered households, and these cities have higher levels of medical care and education (the medical level and education level variables use the registered population). Therefore, both geographic location and population density of cities will affect USDI. The importance of IS still ranks first, indicating that the adjustment of industrial structure is the most important for the urban sustainable development.

### 4.2. Regional Heterogeneity Research

Dividing the data into east, middle, and west for random forest regression further improves the generalization ability of the model, and the performance of the random forest algorithm is better than that of XGboost or MLR (Table 4). Since the random forest model performs better in models 2 and 3, the following studies will exclude model 1.

The article "Using a Random Forest Model to Study the Impact of Local Government-Led Urbanization on Urban Sustainable Development" was published in 2022. Journal: J Environ Public Health.

In model 2, the importance of PD, GR, RED, and LRM in the eastern, mid, and western regions makes heterogeneity (Figure 5). After splitting GR, LRM still shows great heterogeneity. The importance value of the random forest model is obtained by adding noise interference to the OOB. Therefore, the smaller the importance value of the feature, the stronger the noise of the dataset. The strong noise of the variable indicates that the data tend to be randomly distributed in different years. For policy variables, the strong noise indicates that local governments have large changes in policy designation each year. For example, the importance of LRM in the mid is the highest, indicating that the LRM strategies of the midlocal governments are regular. In contrast, the LRM strategies of eastern and western local governments have great volatility. However, due to the large difference in land prices between eastern and western regions, the LRM strategies of eastern and western local governments should be different. The eastern local government maximizes LR by continuously adjusting the LRM strategy, while the western local government cannot misallocate land resources.

AOIE, IS, and PD show great importance in both models, which verifies the conclusion in 4.1. Regarding the analysis of the theoretical mechanism, PD determines the level of education and medical care in the city, IS determines the level of cities' economic development, and AOIE determines the level of wastewater and waste pollution in the city. The local government should focus on improving these three indicators to increase USDI, for example, reducing the number of agreements and industrial land transfers and increasing the AOIE; actively adjusting the industrial structure and improving the level of local economic development; rationally increasing the construction of hospitals and schools in the process of urbanization.

### 4.3. Representative Urban Agglomeration Research

Beijing-Tianjin-Hebei (BTH), Yangtze River Delta (YRD), Pearl River Delta (PRD), and Chengdu-Chongqing (CC) are the four most representative urban agglomerations in China. These four urban agglomerations account for 36.3% of China's population and 47.3% of China's GDP.  Table 5 shows that the generalization ability of the random forest model is improved by choosing the representative urban agglomerations. The performance of the random forest model is still better than XGBoost and MLR.

Figure 6 shows that IS and AOIE have a strong impact on the USDI of the four urban agglomerations, which strengthens the previous results. The GR of these urban agglomerations has a strong impact on the USDI. Due to the strong ability of land resource control, the local governments will adjust LR and LRM strategies to cover excess spending. Therefore, the impact of LRM and LR in these urban agglomerations on USDI is not obvious, but the GR is contrary. The importance of SIFR in BTH and CCCC is obvious, which is different from YRD and PRD. The RED and PD of the four urban circles are stable in both models.

The article "Using a Random Forest Model to Study the Impact of Local Government-Led Urbanization on Urban Sustainable Development" was published in 2022. Journal: J Environ Public Health.

### 4.4. Discussion of Results

From the regression results, IS has the greatest impact on urban sustainable development. Because cities with a high proportion of tertiary industry mean a small proportion of industrial output, there will be fewer emissions of waste gas and wastewater. Therefore, the government should actively adjust the industrial structure to improve the level of sustainable urban development. However, the industry is the foundation of national economic development. Excessively increasing proportion of the tertiary industry will lead to the relocation and loss of manufacturing. Therefore, for cities with a high proportion of industrial output, local governments should focus on improving the output quality and efficiency of industrial enterprises to improve the level of urban sustainable development. The importance of AOIE to urban sustainable development confirms it. Local governments should not continue to increase the number of industrial enterprises through the land resources mismatch but increase output and reduce pollution by providing tax incentives and R&D subsidies for enterprises. Surprisingly, SIFR showed a great impact in BTH and CC and was as important in PRD and YRD as AOIE. Local governments need to work hard to improve the level of urban sustainable development by improving the level of SIFR. However, raising the SIFR level will increase the tax burden for both businesses and residents. Local governments should find a compromise solution to this problem.

The impact of LRM and LR on urban sustainable development is not as important as expected, probably because the intervention of local governments in land supply makes land prices cyclical. The purpose of local government intervention in land supply is to maximize government revenue, which is confirmed by the importance of GR. The importance of LRM and LR gradually increases as the region shrinks. This shows that the local government's land resource allocation strategy is affected by the neighboring cities.

## 5. Conclusions

This paper discusses the impact of government revenue expansion, land resource mismatch, and industrial structure adjustment on sustainable urban development in the process of urbanization. Our research shows that the adjustment of industrial structure and the level of local government income have a great impact on urban sustainable development. The importance of land resources mismatch is stronger in representative metropolitan research. The author believes that land resources mismatch is a measure adopted by local governments to increase the level of income, which is highly cyclical and difficult to detect. The government's influence on sustainable development through land management is reflected in the government revenue.

The article "Using a Random Forest Model to Study the Impact of Local Government-Led Urbanization on Urban Sustainable Development" was published in 2022. Journal: J Environ Public Health.

Urbanization led by local governments will affect sustainable development in many aspects. Local governments will plan land construction after land requisition, including planning the area of industrial, commercial, and residential land, the number of schools and hospitals, public greening, and roads. Land construction planning has different impacts on urban sustainable development. For example, industrial enterprises will cause environmental pollution due to the discharge of waste gas and wastewater; population aggregation will improve the level of medical care and education. Therefore, how local governments plan for land determines the direction of sustainable urban development. Since the reduction in land resources mismatch will reduce the local government revenue, the local government will choose to reduce the expenditure on public services to maintain the speed of economic development. Therefore, the central government should change the promotion incentives and encourage local governments to devote more resources to urban sustainable development. And the central government needs to undertake the corresponding sustainable development construction tasks instead of handing all the tasks to the local governments. This is because the local government adopts a fiscal expansion strategy due to the excess construction tasks. After the central government's incentive mechanism changed, local governments should formulate development strategies according to the industrial structure of the city, not just maximizing the speed of economic development and maximizing government revenue. In the process of industrial transformation and upgrading, the normal operation of the urban economy must be ensured first, and blind and radical strategies should not be adopted.

In addition, local governments should be committed to improving the level of social insurance income in cities, but they should not increase the tax burden on businesses and residents. We think the best way is to let state-owned enterprises take this responsibility. Due to the government's endorsement, state-owned enterprises have advantages over private enterprises in financing and procurement. Therefore, state-owned enterprises are equivalent to enjoying the preferential treatment of market resource allocation. The specific plan is to transfer part of the annual profits of state-owned enterprises to the social insurance fund.

The article "Using a Random Forest Model to Study the Impact of Local Government-Led Urbanization on Urban Sustainable Development" was published in 2022. Journal: J Environ Public Health.

Our study shows that random forest models perform better in government decision-making problems, but how to select variables to measure the level of urban sustainable development more accurately deserves further research. In future research, we will further improve the urban sustainable development index system, and the measurement of land resource mismatch will also adopt a variety of methods.

## Figures and Tables

**Figure 1:** The principle of the random forest model.

**Figure 2:** An example of a local government decision affecting sustainable development.

**Figure 3:** The generalization ability of the three models. (a) Representative model 1, (b) representative model 2, and (c) representative model 3.

**Figure 4:** The importance of variables of the three models. (a) Model 1, (b) model 2, and (c) model 3.

**Figure 5:** The importance of variables of the three models. (a) Corresponding to model 2; (b) corresponding to model 3.

**Figure 6:** The importance of variables of the three models. (a) Corresponding to model 2; (b) corresponding to model 3.

**Table 1:** A simple Nash equilibrium game of local government competition.

Local governments a/b	GDP development	Sustainable development
GDP development	*ρ*_1_+*σ*_1_, *ρ*_1_+*σ*_1_^1^	*ρ*_1_+*σ*_1_, *ρ*_2_+*σ*_2_
Sustainable development	*ρ*_1_+*σ*_1_, *ρ*_2_+*σ*_2_	*ρ*_2_+*σ*_2_, *ρ*_2_+*σ*_2_

*ρ*_1_ and *σ*_1_ corresponding to economic growth mode. *ρ*_2_ and *σ*_2_ corresponding to sustainable development model.

**Table 2:** Composition indicators of USDI.

Indicator	Unit	Connotation	Effects
GDP per capita	RMB	Economic development level	Positive
Green coverage	%	Urban greening level	Positive
Carbon emissions per capita	Ton/p	Energy consumption	Negative
Industrial waste gas emissions per capita	Ton/10000 p	Air pollution	Negative
Industrial wastewater discharge per capita	Ton/p	Water pollution	Negative
Proportion of primary and secondary school teachers	‰	Education	Positive
Proportion of doctors	‰	Medical and health	Positive

**Table 3:** Robustness test of random forest model.

Model	Random forest				XGBoost				MLR
	*R* ^2^		RMSE^*∗*^		*R* ^2^		RMSE		*R* ^2^
	Train	Test	Train	Test	Train	Test	Train	Test	
1	0.913	0.459	0.013	0.030	0.526	0.504	0.027	0.027	0.427
2	0.957	0.704	0.009	0.022	0.540	0.474	0.027	0.029	0.506
3	0.958	0.740	0.009	0.020	0.794	0.519	0.018	0.027	0.508

^*∗*^RMSE is the root mean square error.

The article "Using a Random Forest Model to Study the Impact of Local Government-Led Urbanization on Urban Sustainable Development" was published in 2022. Journal: J Environ Public Health.

**Table 4:** Robustness test of random forest model.

Model	Location	Random forest				XGBoost				MLR
		*R* ^2^		RMSE		*R* ^2^		RMSE		*R* ^2^
		Train	Test	Train	Test	Train	Test	Train	Test	
2	East	0.966	0.803	0.007	0.017	0.893	0.792	0.012	0.018	0.667
	West	0.948	0.690	0.010	0.022	0.779	0.648	0.019	0.023	0.480
	Mid	0.957	0.754	0.008	0.018	0.846	0.682	0.014	0.020	0.467
3	East	0.970	0.825	0.007	0.016	0.902	0.796	0.012	0.018	0.668
	West	0.956	0.759	0.011	0.024	0.900	0.731	0.016	0.022	0.413
	Mid	0.959	0.684	0.008	0.020	0.900	0.680	0.011	0.020	0.442

**Table 5:** Robustness test of random forest model.

Model	Location	Random forest				XGBoost				MLR
		*R* ^2^		RMSE		*R* ^2^		RMSE		*R* ^2^
		Train	Test	Train	Test	Train	Test	Train	Test	
2	BTH	0.982	0.896	0.005	0.011	0.951	0.879	0.009	0.011	0.838
	YRD	0.971	0.839	0.006	0.015	0.902	0.810	0.011	0.017	0.676
	PRD	0.980	0.770	0.006	0.018	0.920	0.903	0.011	0.012	0.767
	CC	0.974	0.847	0.007	0.017	0.924	0.846	0.011	0.017	0.632
3	BTH	0.989	0.913	0.004	0.012	0.953	0.911	0.008	0.010	0.903
	YRD	0.967	0.736	0.008	0.018	0.895	0.766	0.012	0.018	0.555
	PRD	0.979	0.889	0.006	0.014	0.949	0.854	0.009	0.015	0.801
	CC	0.975	0.879	0.007	0.014	0.901	0.827	0.013	0.017	0.733

## Data Availability

All data used to support the findings of this study are included within the article.
